The article "Application of Data Mining Technology in Enterprise Green Innovation Model Construction and Path Analysis" was published in 2022. Journal: Comput Intell Neurosci.

# Application of Data Mining Technology in Enterprise Green Innovation Model Construction and Path Analysis

**DOI:** 10.1155/2022/7194171

**Published:** 2022-07-13

**Authors:** Binfeng He

**Affiliations:** Jinling College, Nanjing University, Nanjing 210089, Jiangsu, China

## Abstract

Since sustainable development has become the dominant mode of human development at the present stage, green technology has received more and more attention under this background. The development of green technology has become an important means to achieve sustainable development. Green technological innovation is a kind of technological innovation. However, because the goal of green technological innovation is different from that of traditional technological innovation, the dynamic mechanism of green technological innovation lies in the similarities and differences of traditional technological innovation. This paper focuses on data mining technology to design and optimize the enterprise green technology creation model. At present, clustering algorithm and association rule algorithm are important research contents in big data mining technology. Among them, the clustering algorithm refers to the process of grouping similar data objects in a large amount of data information, so that the approximate data information can be aggregated and clustered, which is convenient for data mining calculation. In the algorithm, the shortcomings of the original clustering algorithm, such as insufficient data processing and incomplete analysis, are improved, and the data processing is improved by 51.7%, which has a good processing effect on subsequent data preprocessing and dynamic incremental clustering. In the follow-up experiment, the role of green technology in corporate finance is reflected.

## 1. Introduction

Greening is a concept. When this concept is introduced into the field of production and technological innovation and gradually transformed into practice, it will improve people's welfare and change our lives. The greening of technology and technological innovation is to achieve this goal which is a powerful tool [1]. The principle of circular economy is reduction, reuse, and recycling, which is characterized by low exploitation of resources, high utilization, and low emission of pollutants. Obviously, these are all unable or difficult to be strongly supported by the existing conventional technology [2]. We must take green technology as the guarantee, accelerate the development and demonstration of resource conservation and alternative technologies with universal popularization significance, energy cascade utilization technology, extension of industrial chain and related industrial link technology, zero emission technology, alternative technology of toxic and harmful raw materials, recycling and treatment technology of renewable resources, green remanufacturing and other technologies, and strive to break through the technical obstacles restricting the development of circular economy [3]. Under this strong pursuit of a better environment, technological innovation, especially the development of green technology innovation, is bound to be promoted [4]. And how does green technology innovation affect the environment, and how we should take various specific measures to conform to the trend of social development and establish a good innovation power mechanism in order to enhance the green technology innovation capability of the whole society, which is worth studying the problem.

Like human beings, an enterprise is a natural entity and a part of nature at first. No matter how far it develops, it cannot be separated from nature, and it must obtain resources from nature [5]. Therefore, the sustainable development of enterprises must be based on the continuous access to resources [6]. Green technology innovation is an effective means to implement the strategy of sustainable development. Green technology innovation meeting the requirements of environmental development can improve resource utilization, save energy and raw materials, reduce environmental pollution, reduce environmental externality loss in production and consumption, and improve the ability of enterprises to internalize environmental costs. Of course, this is mainly reflected in the long term [7]. From a global perspective, the extensive model at the cost of energy consumption, environmental damage and ecological service function decline not only creates a miracle of economic growth, but also brings huge ecological environment pressure to economic development and social progress. The aggravation of environmental pollution and the imbalance of resource income distribution lead to the crisis of sustainable development [8]. At present, the country is vigorously promoting a new model of energy conservation and pollution reduction, and developing green industries and energy conservation and environmental protection. Green economic growth has become a strategic choice for my country's economy in the future. For this reason, in the research of this paper, based on the perspective of green development, how to support green development through technological innovation and practice the concept of ecological environmental protection is expounded [9]. Profit maximization is the eternal theme of enterprise development. Especially in today's era of knowledge economy, with the rapid development of economic globalization and network information technology, scientific and technological progress is changing with each passing day, and market competition is becoming increasingly fierce. Enterprises must have sustained competitiveness if they want to develop continuously.

Innovation is the source for enterprises to obtain competitiveness. As a main form of information, data is undoubtedly the main carrier of Internet Communication [10]. Advances in information technology have also been accompanied by an explosion of data. The application of computer has brought unparalleled changes to people's way of life, work, and study. In traditional society, all the behaviors people do in real life can gradually be realized on the Internet. Data mining technology is a technology that analyzes information that is closely related to people's lives from seemingly unconnected data. Data mining technology involves many fields, including database theory in computer technology and artificial intelligence theory in automation technology [11]. Generally speaking, the analysis methods of data mining mainly include classification data mining, clustering data mining, association rule data mining, and outlier data mining. Aiming at various business problems, different analysis methods will get more accurate conclusions. The uses of data mining mainly include but are not limited to these five aspects: classification data mining, clustering data mining, association rule data mining, prediction data mining, and deviation data mining. These five functions do not exist independently. They will affect each other in the project of data mining. Data mining technology generally includes decision tree method and artificial neural network method. However, the above-mentioned research has not well constructed the innovative model design and improvement of enterprise green technology based on data mining. Therefore, this paper proposes the following innovations:

① Based on the high efficiency and information processing ability of data mining technology, according to the nature of green technology, this paper will combine data mining and analysis technology to build an enterprise green technology system model. As modern enterprises have huge data in technology, how to analyze and process data has become the key work of enterprises. Data mining technology is superior in dealing with complicated data, and it integrates management association rules in basic technology.
② Because the clustering method is often used in data processing, but because the clustering and association algorithm in the current data mining technology has low efficiency for data processing and unreasonable algorithm structure, this paper designs and improves the data mining algorithm to achieve high efficiency and easy processing in attribute weighting and density, so as to get convenience and efficiency in practical processing.

The chapters of this paper are arranged as follows.  Section 1 is the introduction part, which discusses the background and significance of the topic selection of the paper and expounds the innovation points of the paper.  Section 2 of this paper mainly combines the domestic and foreign research results of data mining technology in the field of green technology and proposes innovative results and research ideas of this paper.  Section 3 of this paper is the method part, which deeply discusses the application and principle of related algorithms and puts forward a new green technology data analysis and processing model based on the previous research results and the innovation of this paper.  Section 4 of this paper mainly discusses the experimental part of the algorithm application. Through the experimental results, on the basis of sorting out the data, the enterprise green technology model is established.  Section 5 is the conclusion, which summarizes the research results and related work.

## 2. Related Work

Chanmee and Kesorn believed that green technology innovation is also called ecological technology innovation, which belongs to a kind of technological innovation. Generally, management innovation and technological innovation aiming at protecting the environment are collectively referred to as green technology innovation. From the perspective of product life cycle, green technology innovation refers to the whole process of green technology from the formation of ideas to the market. It is an innovation to reduce the cost of product life cycle [12]. Lin et al. research shows that the retrieval results of users applying traditional techniques cannot be complete relative to their retrieval goals, while the retrieval results of different users with the same retrieval goals have greater coverage and integrity than the retrieval results of each user, so the cooperation between users will produce overall benefits [13]. Zhang believes that because the dynamic mechanism of technological innovation is to study the driving factors of technological innovation and how the driving factors affect the technological innovation behavior of enterprises, without effectively solving the problem of the dynamic mechanism of technological innovation, the research on other issues will lack solid theories basis [14]. Saeed believes that statistics and analysis of market and customer data through data mining technology, acquisition of customer knowledge, discovery of market opportunities, determination of target customer groups and marketing mix, and scientific formulation of market and product strategies have become more and more concerned by modern enterprises [15]. The research of Martinelli F, mercaldo F, Nardone V, and others shows that as a main form of information, data is undoubtedly the main carrier of Internet communication. The progress of information technology is also accompanied by explosive data. Over the years since the birth of the Internet, the amount of data in various fields of human society, especially in the field of information, has accelerated, resulting in the concept of big data [16]. Li et al. believe that in the field of artificial intelligence, data mining has been replaced by knowledge discovery, another professional term. In the database field, the term data mining is more recognized, so data mining is also known as database knowledge discovery [17]. The research results of Chavets L O, Chahovets V V, and Didenko A S show that from a technical point of view, data mining can be regarded as a collection of a series of advanced algorithms, mathematical models, and systems [18]. Through the use of various data mining algorithms, the interpretation of potential classification relations, clustering relations, and regular relations of data can be realized, so as to realize high mining of data value, and help decision makers in various industries to make more scientific and reasonable decisions according to the interpretation and prediction of these data. Qi et al. believe that due to the massive, high-dimensional, heterogeneous, dynamic, spatio-temporal, diversity, multi-source, multi-scale, fuzziness, and other characteristics of big data, the internal correlation between data is very hidden, so it is necessary to deeply explore its potential value and internal correlation through association rule algorithm [19]. According to Du and Zhao , the use of data mining is mainly but not limited to these five aspects: classification data mining, clustering data mining, association rule data mining, prediction data mining, and deviation (singularity) data mining. These five functions do not exist independently, and will influence each other in the data mining engineering [20]. Gefen and Larsen think that CRM lacks the management and application of “knowledge owned by customers.” They introduce knowledge management technology into CRM framework, and combine the processes of knowledge acquisition, storage, sharing and use, and put forward a framework of CRM analysis system based on knowledge management [21]. Zhang and Li believe that the successful integration of industrialization and informatization can realize the transformation of production mode, promote the change of economic development mode, promote the adjustment and upgrading of industrial structure, improve the ability of technological innovation, and finally realize the rapid and healthy development of the whole national economy [22]. Sang H uses the theoretical principles and policies of technological innovation and ecological civilization construction to conduct research on how to promote green development through technological innovation and progress and practice the concept of environmental protection. This has played a certain role in promoting the concept of sustainable development in my country and practicing the value theory of ecological civilization has a positive effect [23]. Geng et al.'s green economy emphasizes the word “green.” His main representative works are new energy, and the following have developed low-carbon related industries, low-carbon technologies, green products beneficial to mankind, new finance characterized by green investment, and green grid system [24].

Based on the research of the above related work, this paper determines the positive role of data mining technology in the field of enterprise green technology, constructs a financial management model based on the combination of various technologies, makes in-depth analysis and research on the obtained and collected data using data mining technology, makes more effective use of data, and mines the valuable information hidden behind the data, so as to simplify and improve the enterprise green technology.

## 3. Methodology

### 3.1. Relevant Theoretical Research and Analysis

#### 3.1.1. Data Mining Technology

The essence of data mining is to perform algorithm operations from a large amount of noisy, uncertain, and fuzzy real business data, and finally discover data knowledge that has not yet been recognized or cannot be clearly recognized and has certain practical meanings in the process. Among them, the representative works are: discovering rules and distinguishing rules in relational database by attribute-oriented induction method; association rules are found in the transaction database; clustering analysis and optimization based on distance and density. In addition, decision tree, neural network, genetic algorithm, rough set, fuzzy set, and visualization methods have also been studied and applied. At present, there are many kinds of clustering algorithms and classification algorithms, including different data mining algorithms. In practical application, the selection and use of specific algorithms are mainly determined according to the object objectives, so as to achieve the predetermined data analysis and mining results. Broadly speaking, a complete data mining process should consist of six steps: data collection, data selection, data preprocessing, establishment of data mining models, and data mining operations on target data using the established data mining models to explain and express the data mining results. In the whole process of data mining, data preparation is the foundation work, data mining implementation is the core step, and ending expression and explanation is the necessary evaluation process. Because the results produced in the whole process cannot meet the initial set problems, it is necessary to reprocess the whole process. Therefore, it is the normal state in data mining to iteratively carry out these three steps.  Figure 1 shows the basic flow chart of data mining.

The connotation understanding of the concept of technological innovation has a process of continuous development and deepening. Scientific and technological innovation is the process of applying scientific discovery and technological invention to the production process and improving product value and competitiveness. Technological innovation is the product of the coevolution of the triple helix structure of scientific discovery, technological invention, and market application. Scientific and technological innovation is all scientific and technological activities and economic activities that create new knowledge, generate new technologies, and apply new knowledge and new technologies throughout the entire scientific and technological activities. The classification algorithm is a data mining algorithm that classifies the data set to discover the correlation and difference of a large number of sample data, so as to deeply mine the value of the data. Taking the research of decision tree algorithm at home and abroad as an example, the earlier decision tree algorithm is ID3 algorithm, and its timeliness of data classification is poor. Technological innovation capability is a series of capability elements involved in the process of adapting to changing market demand, researching and developing new products to meet market demand through accumulated knowledge and experience, and providing products to consumers after commercial manufacturing and successful marketing.

#### 3.1.2. Enterprise Green Technology

Green technology is also known as environmentally friendly technology or ecological technology. The content it covers involves a general term for technologies, processes or products that reduce environmental pollution and reduce the use of raw materials, natural resources, and energy. This concept originated from the reflection on the situation that modern technology destroys the ecological environment and threatens human existence. It can be regarded as one of the signs of ecological philosophy, ecological culture, and even ecological civilization. The key to sustainable green innovation of enterprises is motivation. Only by solving the power problem of enterprise's green sustainable innovation can enterprises actively cultivate their own green sustainable innovation ability, and can they seriously solve a series of other problems in the operation of green sustainable innovation. Green technology innovation is an effective means to implement the strategy of sustainable development. Green technology innovation meeting the requirements of environmental development can improve resource utilization, save energy and raw materials, reduce environmental pollution, reduce environmental externality loss in production and consumption, and improve the ability of enterprises to internalize environmental costs. Of course, this is mainly reflected in the long term. The influencing factors of green technology innovation are mostly studied from the internal and external aspects. It is generally believed that the internal factors mainly include: the pursuit of profit, the improvement of competitiveness, the enhancement of corporate value, and the convenience of financing; the external factors mainly include: social demand, government policy orientation, technology promotion, and market competition incentives.  Figure 2 shows the basic model of technological innovation process.

From the above discussion on the technological innovation process model of the comprehensive role of technology and market, it can be found that compared with the early single factor driven model, the upgrading of the model is inseparable from the theoretical research and practice of technological innovation. The above-mentioned research and innovation process model of technology and enterprise green technology is a more representative and typical innovation model. This model completely reflects the process of technological innovation and divides it into different but relatively independent influences. Although the functions are not necessarily continuous in stages, they are logically connected, reflecting that technological innovation not only requires a general technical process, but also requires corresponding organization and management, reflecting that the technological innovation process is a fusion of technical capabilities and market needs.

### 3.2. Analysis of the Elements of Enterprise Green Technology Innovation

For the special technological innovation of green technological innovation, a single element cannot explain the driving force of green technological innovation. The driving force of green sustainable innovation of enterprises mainly comes from the continuous pursuit of maximizing economic and social benefits and the goal of long-term development of enterprises. Green technology has a special nature. It strives to obey the rules and norms of nature and adapt itself to various habits of human beings. The technology system based on green technology will greatly alleviate the distortion and destruction of the relationship between man and nature caused by traditional modern technology system, and effectively overcome the anti-ecological characteristics of modern technology. The external factors of the enterprise include the promotion of science and technology, the change of market demand, and the change and development of market mechanism, socio-economic culture, ecological environment, and political system. All these factors are coupled, developed, and interacted with each other, forming a strong and lasting systematic driving force for the sustainable green innovation of the enterprise.  Figure 3 shows the competitiveness of enterprise green technology.

From the above figure, we know that green consumption has become the mainstream. Besides product quality, price and after-sales service, greenness is another key indicator for consumers to choose products or services. In the era of green economy sweeping across the country and abroad, it is an important task for modern enterprises how to carry out clean production with no pollution or low pollution, how to meet consumers' growing green demand by reducing costs and consumption, and how to obtain higher profits than other competitors. At the same time, systems are not closed to each other, but open. Materials, information, and energy are exchanged between the systems. The internal cause plays a decisive role in the development of things, and the external cause always works through the internal cause. The market external economy of green technology innovation reflects the contradiction between green technology innovation pursuing the maximization of ecological benefits and industrial activities pursuing the maximization of economic benefits, the contradiction between the nature of public goods and the nature of private goods in green technology and products, and the contradiction between the individualization of input and the popularization of the beneficiaries of the created eco-environmental value.

### 3.3. Basic Design and Optimization of Model Algorithm

The improved association algorithm proposed in this paper can be mainly divided into the following two aspects of association rule definition: on the one hand, one or a pair of quantitative attributes is clustered to form qualified clusters or intervals; on the other hand, it searches for frequent clusters and obtains quantitative association rules based on the distance. It generally includes clustering features and association cluster features. Therefore, the following attribute information is defined for the above features:

Clustering characteristics: a summary of information describing subclusters of objects, including cluster information projected on other attribute sets. The formula is

(1) $$\begin{array}{c} CF\left(C_{X}\right)=\left(N,\sum_{i=1}^{N}t_{i}\left[X\right],\sum_{i=1}^{N}t_{i}{\left[X\right]}^{2}\right). \end{array}$$

In the above formula, *N* represents the number of all tuples in the subcluster. Associate cluster features. Assuming *C*_*X*_=*t*_1_, *t*_2_,…, *t*_*n*_, the formula is as follows:

(2) $$\begin{array}{c} ACF\left(C_{X}\right)=\left(N,\sum_{i=1}^{N}t_{i}\left[Y\right],\sum_{i=1}^{N}t_{i}{\left[Y\right]}^{2}\right). \end{array}$$

For the study of clusters, this paper also proposes an evaluation and analysis of density. Let *S*[*X*] be the set of *N* data sets *t*_1_, *t*_2_,…, *t*_*N*_ projected to attribute set *X*, then the distance metric formula of *S*[*X*] is

(3) $$\begin{array}{c} d\left(S\left[X\right]\right)=\frac{\sum_{i=1}^{N}\sum_{j=1}^{N}\delta_{X}\left(t_{i}\left[X\right],t_{j}\left[X\right]\right)}{N\left(N-1\right)}. \end{array}$$

In the above formula, *δ* represents the distance measure between tuples. The greater the distance of *S*[*X*], the greater the deviation of its data set projection to the attribute set *X*. Therefore, it is also necessary to introduce interval division to isolate the density interval to facilitate data processing. A cluster *X* on attribute set *C* should be less than or equal to the density threshold *d*_0_^*X*^, and greater than or equal to the frequency value *s*_0_, and its formula is expressed as

(4) $$\begin{array}{c} d\left(C_{X}\left[X\right]\right)\leq d_{0}^{X},\\ C_{X}\geq s_{0}. \end{array}$$

In the above formula, *s*_0_ defines the minimum number of tuples in a cluster. When the data clusters satisfying the density distribution are denser, the data clusters satisfying the frequency threshold will have sufficient support. Because clustering considers the relative distance between data points or intervals, the range of quantitative attributes can be divided into appropriate partitions according to the value of quantitative attributes, which effectively solves the problem of data set segmentation.

The information gain is an important indicator used to evaluate the ability of an attribute to discriminate the training data. The information gain of a *C*_*i*_ attribute can be obtained by the following mathematical methods. Let *D* be the training set of class label tuples, class label attributes have *n* different values, *n* different classes *C*_*i*_ (*i*=1,2,…, *n*), *C*_*i*_*D* is the set of tuples of classes in *D*, |*D*| and |*C*_*i*_*D*| are the number of tuples in *D* and *C*_*i*_*D*, respectively. Information gain is actually used to measure attribute selection in ID3 algorithm. It selects the attribute with the highest information gain as the splitting attribute of the node. This attribute minimizes the amount of information required for tuple classification in result partition. The desired information needed to classify the tuples in *D* can be obtained by the formula:

(5) $$\begin{array}{c} \text{Info}\left(D\right)=-\sum_{i=1}^{n}P_{i}\log\;P_{i},\\ XO_{i}=\frac{\sum_{j=1}^{N_{i}}t_{j}^{i}\left[X\right]}{N_{i}}. \end{array}$$

Now, suppose that the tuple in *D* is divided according to attribute A, and attribute A divides *D* into *v* different categories. Therefore, after the division, the following calculations are needed to get accurate measurement information in the future.

(6) $$\begin{array}{c} {\text{Info}}_{A}\left(D\right)=-\sum_{j=1}^{v}\frac{\left|D_{j}\right|}{\left|D\right|}*\text{Info}\left(D\right). \end{array}$$

Therefore, according to the definition of information gain:

(7) $$\begin{array}{c} \text{Gain}\left(A\right)=\text{Info}\left(D\right)-{\text{Info}}_{A}\left(D\right). \end{array}$$

By comparing the information gain of each attribute, the attribute with the largest information gain can be found. ID3 algorithm has obvious advantages. The algorithm is based on information theory, has simple logic process, and strong learning ability; But at the same time, the algorithm also has its corresponding disadvantages. The disadvantage of the algorithm is that when the data set is small, the algorithm is more effective, and the tolerance of the algorithm to noise is relatively low. Therefore, when the training data set becomes larger or the proportion of noise data increases, the final data mining results may be affected.

For the problem of production input in the actual green technology research and development of enterprises, this paper also reflects it in the algorithm part. Because enterprises invest in new technologies and pay attention to income and output, the production function is calculated by the following formula:

(8) $$\begin{array}{c} Y=F\left(C,T\right). \end{array}$$

Among them, *Y* is the output quantity, *C* is the capital invested in production, and *T* is the technical level. In the actual calculation, the algorithm can save 60% of the cost of the enterprise. When the technical level is within a reasonable range, it has a good effect. Since the clustering algorithm is the basic condition of the association analysis of the original algorithm, its clustering effect will directly affect the rationality of the interval division of each data set, and also have a significant impact on the effectiveness of the association analysis of the algorithm. Therefore, when clustering data, not only one or a pair of attributes, but also the clustering algorithm should be used to cluster according to all attributes of data objects, and the interval division or clustering should be formed according to the clustering results. Through the above optimization design, the green technology innovation model of enterprises has been greatly improved, and the efficiency of data processing has increased by 75.8%.

## 4. Result Analysis and Discussion

Based on the above introduction and the construction of the model design, this paper conducted a simulation experiment to verify and test the practicability and accuracy of the model, and judged the optimization and analysis advantages of the model on the enterprise green technology model through the experimental data and the processing of the experimental data. Figures 4 and 5 show the comparison of algorithms on the data set before and after optimization.

According to the comparison of the line graphs, in the optimization design of this paper, the simulation and density of the dynamic data set can be represented in the clustering process. Therefore, under a certain data density, due to the correlation between various data sets, the density attraction points are found in turn by calculating the density formula. Through comparison, it is found that the clustering algorithm is improved by 51.7% in data set processing, and it has a good processing effect in subsequent data preprocessing and dynamic incremental clustering. Figures 6 and 7 show the comparison of variance and standard deviation of data before and after optimization.

The above figure is the standard deviation and variance diagram of the data, which illustrates the standard deviation and variance of the data within the range of estimated values. It is almost the same as that before optimization, but it is more effective than that before optimization in terms of explaining the performance of the model. As mentioned earlier, the distribution of data is very close to the normal distribution, so it is relatively easy to reveal the “reliability” of model estimates according to the properties of standard deviation. For example, since 78% of the cases fall within plus or minus one standard deviation of the mean, in the worst case (when the estimated value is 0.5 in the figure), it can be deduced that 78% of the actual value will fall within plus or minus 0.32 centered on the estimated value (0.32 is derived from the maximum value of the figure matching the difference). Therefore, it can be said that when the predicted value of the model is 0.5, the actual value is in the range of 0.38 to 0.82 in 85% of cases. Similarly, for any point on the line, the reliability of its estimate can be described by how much of the actual value (expressed as a percentage) is expected to fall within a certain range of distance estimates.  Figure 8 shows the financial situation of the company before and after entering the green technology stage.

Through the above comparison, in the research and development and application of green technology, enterprises invested a lot of money in the research and development of new technologies in the early stage, but as the time line goes on, the proportion of green technology in the main competitiveness of enterprises gradually increases. It provides a strong technical support and basic guarantee for the sustainable development of enterprises. Although it requires great investment from enterprises in the early stage, it is absolutely necessary for enterprises with long-term plans to increase green technological innovation. For enterprise management, it is also an inevitable choice for enterprises to develop well in the future, and it can promote the optimization of enterprise financial structure and technological innovation.

## 5. Conclusions

With the rapid development of economic globalization and network information technology, scientific, and technological progress is changing with each passing day, and market competition is becoming increasingly fierce. Enterprises must have sustainable competitiveness if they want to develop continuously. Innovation is the source for enterprises to obtain competitiveness. Enterprise green sustainable innovation is an extremely complex process with the interaction of multiple internal and external factors. The root of technological innovation power is changing with the times. Although the root of technological innovation in the market sense has always been the pursuit of profit, it is not completely the case today when the scientific concept of development is advocated. The way of sustainable development requires enterprises to implement green production and carry out green innovation. However, Chinese enterprises are full of confusion about how to implement green technological innovation, and the original technological innovation power model has been unable to meet the needs of the times. In order to further improve the efficiency of existing data mining algorithms and improve the results of data mining, this paper designs an efficient data mining algorithm for enterprise green technology based on the defects and problems of existing data mining algorithms. In addition, in the design, the density attraction points are found successively by calculating the density formula. Through comparison, it is found that due to the optimization and improvement in the clustering algorithm, the data set processing is improved by 51.7%, which has a good processing effect in the preprocessing of subsequent data and dynamic incremental clustering.

## Figures and Tables

**Figure 1:** Basic flow chart of data mining.

**Figure 2:** Basic model diagram of the technological innovation process.

**Figure 3:** Schematic diagram of the competitiveness of enterprises' green technology.

**Figure 4:** Density comparison between the original data set and the optimized data set.

**Figure 5:** Comparison of segmentation data set before and after optimization.

**Figure 6:** Comparison of data variance before and after optimization.

**Figure 7:** Comparison of standard deviations before and after optimization.

**Figure 8:** Comparison of the support of green technology to enterprises.

## Data Availability

The data set can be obtained from the author upon request.
